# Comprehensive Assessment of Dermatologic and Dysmorphic Manifestations in Patients With Down Syndrome

**DOI:** 10.1111/srt.70077

**Published:** 2024-10-07

**Authors:** Gökhan Kaya, Ceren Alavanda

**Affiliations:** ^1^ Department of Dermatology Ministry of Health Nizip State Hospital Gaziantep Turkey; ^2^ Department of Medical Genetics Ministry of Health Van Training and Research Hospital Van Turkey

**Keywords:** comprehensive health management, dermatological care, dermatological findings, Down syndrome, genetics, trisomy 21

## Abstract

**Background:**

Down syndrome (DS), a common chromosomal anomaly caused by trisomy of chromosome 21, is characterized by a broad spectrum of phenotypic characteristics across multiple organ systems, including cardiac defects and leukemia. Dermatological findings are prevalent among individuals with DS; however, these issues are frequently underrecognized and inadequately researched, resulting in a significant gap in the provision of comprehensive healthcare strategies. Given the increased life expectancy of patients with DS and delayed manifestation of many dermatoses, physicians are increasingly encountering dermatological findings in this population.

**Objective:**

This study aimed to assess the prevalence and types of dermatological findings in individuals with DS, compare them with those in a control group, and emphasize the necessity of incorporating dermatological evaluations into routine health monitoring.

**Methods:**

This prospective cross‐sectional study was conducted from June 2023 to June 2024 and involved 100 genetically confirmed individuals with DS and 100 age‐ and sex‐matched controls. Comprehensive demographic, clinical, and karyotype data were collected for the DS group, and all the participants underwent detailed morphological evaluations.

**Results:**

The DS group had a mean age of approximately 6.37 years, whereas the controls were around 7 years old, with no significant differences in age or sex distribution between the groups. Karyotype analysis showed that trisomy 21 was present in 92% of the cases, mosaicism in 6%, and translocation in 2%. Common dermatological findings in the DS group included xerosis cutis (49%), thin and sparse hair (48%), dental caries (34%), delayed tooth eruption (28%), nail dystrophy (25%), fissured tongue (23%), and cheilitis (18%). Significant differences were noted in the prevalence of scabies, bacterial infections, and café au lait macules between the DS and control groups (*p* < 0.01). Dysmorphic findings in the DS group included epicanthal folds (97%), upslanted palpebral fissures (97%), brachycephaly (91%), and single transverse palmar crease (89%). Significant gender differences were noted in the prevalence of brachycephaly and the sandal gap (*p* < 0.01).

**Conclusions:**

This study highlights the importance of regular dermatological care in enhancing the health management and quality of life of individuals with DS due to the prevalence and variability of dermatological conditions.

**Abbreviations**
AA: Alopecia areata
APP: amyloid precursor protein
CALM: Café‐au‐lait macules
CTA: Congenital temporal triangular alopecia
DS: Down syndrome
FISH: Fluorescence in situ hybridization
HS: Hidradenitis suppurativa
IFN: Interferon
ISCN: International System for Human Cytogenomic Nomenclature
MMPs: Matrix metalloproteinases
SPSS: Statistical Package for the Social Sciences
TIMPs: Tissue inhibitors of metalloproteinases

## 1 Introduction

Down syndrome (DS), also known as trisomy 21, was first described by British physician John Langdon Down in 1866 [1]. Jerome Lejeune and Patricia Jacobs' landmark research in 1959 identified the cause of DS as trisomy of chromosome 21, a chromosomal anomaly characterized by full or partial extra genetic material on chromosome 21. This leads to pronounced intellectual disability and distinct dysmorphic and phenotypic traits [2]. Epidemiologically, DS occurs in approximately one per 1000 live births, with affected individuals typically aged 50−60 years [3]. Regional studies in Türkiye have reported DS prevalence rates of approximately 0.949 per 1000 live births in Denizli over 16 years [4] and 1.387 per 1000 births in Ankara [5].

Research led by Antonarakis et al. further detailed the structural variations in chromosome 21, including trisomy, mosaicism, and translocation, and elucidated their effects on physical and cognitive development. These insights are crucial for developing targeted therapies for DS [6]. DS is characterized by a spectrum of intellectual and physical developmental challenges, and distinctive facial dysmorphisms apparent from birth. This disorder affects various organ systems, leading to issues in the musculoskeletal, neurological, and cardiovascular systems, such as postural deficits, muscle hypotonia, and congenital heart anomalies. There is also a higher occurrence of conditions such as hypothyroidism, autoimmune disorders, and early‐onset Alzheimer's disease in this population [7]. Chronic dermatological and mucosal conditions are common complications in DS patients.

Despite the prevalence of such issues, literature often underreports detailed examinations of the dermatological and dysmorphic features of DS. Commonly described conditions include xerosis, seborrheic dermatitis, alopecia, and atopic dermatitis. Frequently noted dysmorphic features include epicanthal folds, upslanted palpebral fissures, and brachycephaly [8]. Oral mucosal manifestations such as cheilitis, geographic tongue, and fissured tongue are common and compounded by heightened susceptibility to periodontal diseases and orofacial candidiasis, exacerbated by immunological deficiencies, particularly thymus‐dependent function, and metabolic disorders such as diabetes [9]. Recent studies indicate that 56% of young adults with DS report skin issues [10], and the prevalence of dental anomalies ranges from 50.47% to 95.52% [11].

This study aimed to conduct an extensive analysis of dermatological and dysmorphic findings in individuals with DS and in healthy controls. Including a control group enabled objective comparative assessments, enhancing the understanding of the impact of these manifestations on overall health management and quality of life. Such comprehensive evaluations are instrumental in developing health strategies to improve the quality of life of individuals with DS significantly.

## 2 Materials and Methods

### 2.1 Study Design and Setting

This prospective cross‐sectional study was conducted from June 2023 to June 2024 at the Dermatology Clinic of Gaziantep Nizip State Hospital and the Medical Genetics Department of Van Training and Research Hospital. The primary aim was to compare dermatological findings in individuals with genetically confirmed DS across various age groups. Dermatological assessments were carried out by two separate teams of healthcare professionals. At the Dermatology Clinic of Gaziantep Nizip State Hospital, a certified dermatologist conducted physical examinations and documented all dermatological findings using standardized clinical criteria. In Van, patients were evaluated by a medical geneticist at the Medical Genetics Department, with any diagnostic uncertainties resolved through consultation with the dermatology department.

### 2.2 Ethical Considerations

The study was approved by the Ethics Committee of Van Training and Research Hospital (approval number: 2023/20‐07). Informed consent was obtained from all participants or their legal guardians in accordance with the ethical standards of the 1964 Helsinki Declaration and its later amendments.

### 2.3 Participants

This study included 100 individuals diagnosed with DS and confirmed by karyotyping. Additionally, 100 control subjects without DS were included, ensuring that each control was age‐ and sex‐matched to a DS participant, all of whom were examined at a dermatology clinic. Both the DS and control groups were stratified into four age categories for comprehensive analysis: infants (0–1 year), children (1–12 years), adolescents (12–18 years), and adults (18 years and older).

### 2.4 Data Collection and Clinical Assessment

Comprehensive demographic, clinical, and dysmorphic data, including age, sex, height, and weight were collected from all participants. Each participant underwent thorough dermatological assessments and necessary diagnostic procedures such as dermoscopy and skin biopsy to clarify diagnoses. Personalized treatment recommendations were then formulated based on the individual findings, ensuring tailored management for each participant. All assessments were conducted at a single time point during the participants' initial clinic visits within the study period, which lasted from June 2023 to June 2024. Although some patients continued to visit dermatology outpatient clinics for follow‐up evaluation and treatment after this period, these additional findings were recorded as part of routine clinical care and were not included in the study outcomes due to the cross‐sectional design of the study.

### 2.5 Karyotyping

Karyotype analysis was conducted on G‐banded metaphase chromosomes following a standard protocol with a resolution of 450–500 bands. Twenty‐five metaphases were counted for each patient and at least five metaphases were analyzed. For mosaicism, at least 100 metaphases were counted, and interphase fluorescence in situ hybridization (FISH) was performed using a new blood sample. Results were reported according to the International System for Human Cytogenomic Nomenclature (ISCN 2020) [12].

### 2.6 Statistical Analysis

Before data collection, power analysis was performed to ensure that the study had sufficient power (80%) to detect significant differences at the 5% alpha level. Data analysis was performed using the IBM Statistical Package for the Social Sciences (SPSS) Statistics software (version 25.0). Descriptive statistics were used to summarize demographic and clinical characteristics. Comparisons across the defined age groups were conducted using chi‐square tests for categorical variables and ANOVA for continuous variables, with a significance threshold set at *p* < 0.05.

## 3 Results

### 3.1 Demographic and Anthropometric Data

This study examined 100 individuals diagnosed with DS confirmed by karyotyping, and 100 age‐ and sex‐matched controls. Participants were stratified into four age categories: infants (0–1 year), children (1–12 years), adolescents (12–18 years), and adults (18+ years). The gender distribution was 54% females (*n* = 54) and 46% males (*n* = 46). In the DS group, the average age was 76.49 ± 80.82 months (approximately 6.37 years), ranging from 1 to 396 months (up to 33 years). The mean height was 101.77 ± 35.24 cm, the mean weight was 25.41 ± 22.44 kg, and the mean BMI was 19.40 ± 7.14 kg/m^2^. The mean age of the control group was 83.90 ± 80.38 months (approximately 7 years), ranging from 1 to 372 months (up to 31 years), with the same gender distribution as the DS group. Statistical analysis revealed no significant differences in age (*p* = 0.516) or sex distribution (*p* = 1.0) between groups (Table 1).

**TABLE 1:** Demographic and anthropometric data of DS and control group.

Variable	DS group (Mean ± SD) (*n* = 100)	Control group (Mean ± SD) (*n* = 100)	*p* value
Age (months)	76.49 ± 80.82	83.90 ± 80.38	0.516
Height (cm)	101.77 ± 35.24	Not reported	—
Weight (kg)	25.41 ± 22.44	Not reported	—
BMI (kg/m^2^)	19.40 ± 7.14	Not reported	—
Female (%)	54	54	1.0
Male (%)	46	46	1.0

Abbreviation: DS, Down syndrome.

The demographic and anthropometric characteristics of the study participants are summarized, confirming that the DS and control groups were well matched for age and sex, with no significant differences observed, ensuring the comparability of the groups.

### 3.2 Genetic Findings in the DS Group

Karyotype analysis of the DS group showed that the most common types were 47, XX+21 (43%), and 47, XY+21 (49%), indicating regular trisomy 21. While 46, XX/47, XX+21 and 46, XY/47, XY+21 mosaicisms accounted for 4% and 2%, respectively, translocation type 46, XY, +21, der(21;22)(q10;q10) represented 2% (Table 2).

**TABLE 2:** Genetic findings in the DS group.

Karyotype	Percentage (%)	Count (*n*)
47, XX+21	43	43
47, XY+21	49	49
46, XX/47, XX+21 (Mosaic)	4	4
46, XY/47, XY+21 (Mosaic)	2	2
46, XY, +21, der(21;22)(q10; q10) (Translocation)	2	2

Abbreviation: DS, Down syndrome.

The genetic diversity within the DS population is evident, with regular trisomy 21 being the most common karyotype. Variations such as mosaicism and translocations, though less frequent, highlight the necessity of detailed genetic analysis in clinical assessments of DS.

### 3.3 Dysmorphic Findings

Several dysmorphic features were observed in the DS group. The most common were epicanthal folds and upslanted palpebral fissures, each present in 97% of individuals. Brachycephaly was noted in 91% of cases, and a single transverse palmar crease was found in 89% of cases. A flat nasal bridge was reported in 79%, while dysplastic ears and protruding tongues were observed in 75% and 72% of individuals, respectively. Gender‐specific differences were evident in certain features. Brachycephaly was significantly more prevalent in males than in females (*p* = 0.045). Similarly, the sandal gap was significantly more common in males than in females (*p* = 0.004). However, other features such as the epicanthal fold, single transverse palmar crease, flat nasal bridge, dysplastic ears, and protruding tongue showed no statistically significant gender differences (all *p* > 0.05). The analysis also included the stratification of dysmorphic findings across four age categories infants, children, adolescents, and adults. No significant age‐related differences were noted, suggesting that these dysmorphic features are consistent across age groups in individuals with DS (Table 3).

**TABLE 3:** Prevalence of dysmorphic findings in DS group.

Dysmorphic finding	Female (%) (*n* = 54)	Male (%) (*n* = 46)	Total (%) (*n* = 100)	*p* value
Epicanthal fold	97.8	96.3	97.0	>0.05
Upslanted palpebral fissures	100.0	94.4	97.0	—
Brachycephaly	84.8	96.3	91.0	**0.045**
Single transverse palmar crease	91.3	87.0	89.0	>0.05
Flat nasal bridge	76.1	81.5	79.0	>0.05
Dysplastic ear	73.9	75.9	75.0	>0.05
Protruding tongue	71.7	72.2	72.0	>0.05
Small nose	65.2	57.4	61.0	>0.05
Sandal gap	43.5	72.2	59.0	**0.004**
Small ear	58.7	53.7	56.0	>0.05
Short broad neck	47.8	55.6	52.0	>0.05
Protruding abdomen	56.5	46.3	51.0	>0.05
Clinodactyly	45.7	50.0	48.0	>0.05
Small mouth	47.8	42.6	45.0	>0.05
Fissured tongue	43.5	35.2	39.0	>0.05
Flat nipple	21.7	25.9	24.0	>0.05
Increased nuchal skin fold	10.9	11.1	11.0	>0.05
Strabismus	13.0	5.6	9.0	>0.05
Refractive errors	4.3	3.7	4.0	>0.05
Umbilical hernia	4.3	1.9	3.0	>0.05

Abbreviation: DS, Down syndrome.

Significant differences were found in brachycephaly and sandal gap, both more prevalent in males, while other dysmorphic features were uniformly distributed across genders, reflecting the consistent presentation within the DS population.

Bold values statistically significant parameters less than *p* < 0.05.

### 3.4 Dermatological Findings

In the present study, various dermatological conditions were observed in individuals with DS. The most common findings were xerosis cutis (49%), thin and sparse hair (48%), and dental caries (34%). Notably, only 3% of the patients in the DS group exhibited no dermatological findings.

Significant differences were found between the DS and control groups under several conditions. Xerosis cutis was significantly more prevalent in the DS group (49%) compared to the control group (3%) (*p* < 0.0001). Delayed tooth eruption and fissured tongue were also more common in the DS group, with both conditions showing significant differences (*p* < 0.0001).

Café au lait macules (CALM) were observed more frequently in the DS group (15%) compared to the control group (4%) (*p* = 0.0008). Additionally, bacterial infections were notably more prevalent in the DS group (11%) than in the control group (1%) (*p* = 0.003). In contrast, scabies was found more frequently in the control group (18%) than in the DS group (4%) (*p* = 0.002). Moreover, vascular conditions such as cutis marmorata, livedo reticularis, and acrocyanosis were significantly more prevalent in the DS group (17%) compared to only 1% in the control group (*p* < 0.001).

Beyond the primary findings detailed in Table 4, additional dermatological conditions identified among individuals with DS either highlighted specific challenges faced by this population or were observed at rates comparable to those of the control group, enhancing our understanding of the dermatological profile of DS.

**TABLE 4:** Prevalence of dermatological findings in DS and control groups.

Dermatological finding	DS group (%)	Control group (%)	*p* value
Xerosis cutis	49	3	**<0.0001**
Thin and sparse hair	48	0	—
Dental caries	34	0	—
Delayed tooth eruption	28	1	**<0.0001**
Nail dystrophy	25	0	—
Fissured tongue	23	2	**<0.001**
Cheilitis	18	0	—
Scabies	4	18	**0.002**
Bacterial infections	11	1	**0.003**
Fungal infections	10	6	>0,05
Café au lait macules	15	4	**0.0008**
Alopecia areata	3	7	>0.05
Acanthosis nigricans	3	1	>0.05
Seborrheic dermatitis	6	7	>0.05
Acne vulgaris	4	7	>0.05
Fungal infections	10	6	>0.05
Viral infections	3	7	>0.05
Vitiligo	3	6	>0.05
Atopic dermatitis	6	3	>0.05
Cutis marmorata, livedo reticularis, and acrocyanosis	17	1	**<0.001**
Tooth anomalies	22	0	**—**
Hemangioma	6	3	>0.05
Congenital temporal Triangular alopecia	7	0	—

*Note*: Conditions with nonsignificant *p* values or marked with “−” were not statistically significant, likely due to similar occurrence rates in both groups or limitations in sample size. Regular dermatological evaluations are essential for managing these distinct skin health issues in individuals with DS.

*Note*: *p* values < 0.05 indicate significant differences between the DS group and controls, while *p* values > 0.05 suggest no significant difference or potential sample size limitations. “‐” indicates no statistical analysis was performed.

Abbreviation: DS, Down syndrome.

Notable dermatological differences between individuals with DS and controls include a significantly higher prevalence of xerosis cutis, delayed tooth eruption, fissured tongue, and CALM in the DS group, as indicated by their *p* values. Marked disparities are also evident in the rates of bacterial infections and scabies.

Bold values statistically significant parameters less than *p* < 0.05.

#### 3.4.1 Unique to DS Group

Postinflammatory hyperpigmentation (5%), early hair graying (3%), miliaria rubra (1%), anetoderma (8%), nevus depigmentosus (3%), keratosis pilaris (13%), callus formation (8%), palmoplantar keratoderma (6%), hypertrichosis (2%), striae (6%), Mongolian spots (12%), syringoma (3%), calcinosis cutis (1%), congenital temporal triangular alopecia (CTA) (7%), nail dystrophy (25%), postoperative scars (9%), lichen striatus (1%), pityriasis rosea (3%), burn scars (3%), hidradenitis suppurativa (HS) (1%), acrokeratosis verruciformis of Hopf (1%), nummular dermatitis (1%), and angiokeratoma (1%).

#### 3.4.2 Common Conditions

Hemangiomas (6% in DS vs. 3% in controls), urticaria (2% in both groups), pilonidal sinus (1% in both groups), seborrheic dermatitis (6% in DS vs. 7% in controls), acne vulgaris (4% in DS vs. 7% in controls), fungal infections (10% in DS vs. 6% in controls), viral infections (3% in DS vs. 7% in controls), vitiligo (3% in DS vs. 6% in controls), and atopic dermatitis (6% in DS vs. 3% in controls) were also noted in both groups, but there were no significant statistical differences, suggesting that these conditions occur at similar rates or that variability limits the detectability of a true effect.

Table 5 presents a comparison of various dermatological conditions between male and female individuals with DS. Significant gender differences were observed in conditions such as xerosis cutis, bacterial infections, CALM, fissured tongue, scabies, cutis marmorata, livedo reticularis, acrocyanosis, and delayed tooth eruption. A categorized and photographically illustrated representation of various dermatological findings is depicted in the subsequent figures (Figures 1, 2, 3, 4, 5, 6).

**TABLE 5:** Comparison of dermatological findings by gender.

Dermatological finding	Female (%) (*n* = 54)	Male (%) (*n* = 46)	Total (%) (*n* = 100)	*p* value
Xerosis cutis	52.2	46.3	49.0	**<0.0001**
Palmoplantar keratoderma	6.0	6.0	6.0	>0.05
Atopic dermatitis	6.0	6.0	6.0	>0.05
Keratosis pilaris	13.0	13.0	13.0	>0.05
Bacterial infections	8.7	13.0	11.0	**0.047**
Café au lait macules	10.9	18.5	15.0	**0.009**
Fissured tongue	21.7	24.1	23.0	**0.006**
Scabies	2.2	13.0	7.7	**0.047**
Cutis marmorata, livedo reticularis, and acrocyanosis	17.4	1.9	10.0	**<0.001**
Delayed tooth eruption	34.8	22.2	28.5	**<0.001**
Alopecia areata	4.3	3.7	4.0	>0.05
Seborrheic dermatitis	2.2	3.7	3.0	>0.05
Fungal infections	6.5	13.0	10.0	>0.05
Viral infections	4.3	8.7	6.5	>0.05
Vitiligo	4.3	7.4	5.8	>0.05
Hemangioma	10.9	3.7	7.0	>0.05
Acanthosis nigricans	2.2	1.9	2.0	>0.05
Diaper rash	6.5	1.9	4.5	>0.05
Urticaria	4.3	3.7	4.0	>0.05
Pilonidal sinus	0.0	2.2	1.0	>0.05
Acne vulgaris	0.0	9.3	4.5	>0.05

The prevalence of various dermatological conditions among individuals with DS, categorized by gender, reveals significant differences in xerosis cutis, bacterial infections, CALM, fissured tongue, scabies, cutis marmorata, and delayed tooth eruption.

Bold values statistically significant parameters less than *p* < 0.05.

**FIGURE 1:** Oral manifestations in individuals with DS. (a) Physical examination of a patient with DS revealed inflammatory changes, including redness, soreness, and ulceration on both commissures, likely associated with underlying immune defects, infections, and nutritional deficiencies. (b) Dental examination of a patient with DS reveals multiple orofacial anomalies, including enamel hypoplasia, discoloration, dental caries, and tooth malalignment. These anomalies are linked to disruptions in cellular proliferation during dental lamina and tooth bud development and are driven by complex genetic, epigenetic, and environmental factors. (c) Dental examination of a patient with DS revealed extensive carious lesions characterized by significant discoloration, enamel erosion, and decay. These dental issues are likely exacerbated by challenges such as limited access to dental care, poor dietary choices, use of medications for upper airway infections, inadequate oral hygiene, and insufficient parental support. (d) Physical examination of a patient with DS revealed a fissured tongue characterized by prominent grooves and cracks on the dorsal surface of the tongue. This condition is often associated with macroglossia and a small oral cavity commonly seen in individuals with DS, leading to chronic irritation. DS, Down syndrome.

**FIGURE 2:** Inflammatory and infectious skin conditions in DS. (2) Folliculitis presenting as multiple small, erythematous papules on the chest and abdomen of a DS patient, consistent with inflammation of the hair follicles, commonly due to bacterial infections such as streptococci or fungal infections like malassezia. Often requiring differentiation from abdominal HS, folliculitis is typically more superficial, less painful, and does not involve chronicity, scarring, or sinus tract formation. (b) An atypical localization of hidradenitis suppurativa on the abdomen, likely influenced by obesity and mechanical stress factors, consistent with Hurley stage I. (c) Physical examination of a DS patient revealed multiple erythematous papules and excoriations on the chest and abdomen, indicative of a scabies infestation caused by Sarcoptes scabiei. The patient's low immunity, cognitive impairment associated with DS, and scabies outbreak in our region likely contributed to the development of the infestation. (d) Physical examination revealed widespread verruca vulgaris on the plantar foot, marked by rough raised lesions caused by common benign HPV subtypes, which are more resistant to treatment than warts elsewhere on the skin. DS, Down syndrome.

**FIGURE 3:** Chronic inflammatory disorders and keratinization abnormalities in DS. (a) Lichen striatus, a self‐limiting benign dermatosis, presenting in a DS patient with a linear configuration along the length of the right lower extremity. The distribution of skin lesions along Blaschko's lines warrants consideration of differential diagnoses, such as linear psoriasis and inflammatory linear verrucous epidermal nevus, particularly in patients with DS. (b) In a patient with DS presenting with pruritic, coin‐shaped, erythematous, and eczematous plaques on the back, the initial differential diagnosis included common dermatoses such as tinea corporis or allergic contact dermatitis; however, nummular dermatitis was confirmed based on the patient's history and dermoscopic findings. (c) Palmoplantar keratoderma, characterized by excessive epidermal thickening of the palms and soles, in a patient with DS, developing after early childhood and becoming more common with age. (d) A DS patient with dry skin and a “plucked chicken skin” appearance on the abdomen was diagnosed with xerosis cutis and keratosis pilaris, conditions associated with impaired skin barrier function, increased risk of atopy, and skin infections. DS, Down syndrome.

**FIGURE 4:** Hair and nail findings in children with DS. (a) A child with thin and sparse hair, possibly indicative of an underlying condition affecting hair density, such as hypothyroidism and trace element deficiency, which are often observed in DS. (b) Congenital temporal triangular alopecia, a rare, circumscribed, noncicatricial, and noninflammatory type of alopecia, presents as a distinct triangular area of hair loss at the temple in a patient with DS. During diagnosis, it is important to exclude other conditions such as alopecia areata and aplasia cutis, and to keep in mind the increased prevalence of autoimmune‐related alopecia areata in this population. (c) Early‐onset of graying hair, suggesting premature canities that could be linked to deficient DNA repair mechanisms, leading to accelerated aging along with other health conditions associated with DS. (d) Nail dystrophy, characterized by irregularities in texture and discoloration, is commonly observed in various dermatological conditions, including proximal subungual onychomycosis, inflammatory skin diseases, and environmental factors, in patients with DS. DS, Down syndrome.

**FIGURE 5:** Structural Abnormalities in Individuals with DS. (a) Acrokeratosis verruciformis of Hopf in a patient presenting with verrucous papules and flat‐topped keratotic plaques on the dorsum of the hands. This autosomal dominant genodermatosis, linked to a defect in the ATP2A2 gene on chromosome 12q24, typically develops in early childhood and follows a benign but chronic course, without spontaneous remission. Despite its genetic nature, no similar findings were observed in this patient's family members. Although this condition may not be the first to be considered in this patient group, differential diagnoses should include flat warts, seborrheic keratosis, stucco keratosis, epidermodysplasia verruciformis, and Darier disease. (b) Physical examination of a patient with DS revealed a well‐circumscribed pigmented macule on the back, ranging from light to dark brown, that developed after birth. Solitary café‐au‐lait macules are common and generally benign in the general population, but multiple CALMs may indicate underlying genetic syndromes, such as neurofibromatosis (NF1, NF2) or McCune‐Albright syndrome. (c) Physical examination of a patient with DS revealed multiple, scattered, white to skin‐colored papules with central protrusion on the anterior left chest wall, diagnosed as primary anetoderma, with no history of skin disease before the development of these lesions. Primary anetoderma may result from loss of elastic tissue due to defective synthesis, increased elastolytic enzymes, or autoimmune destruction; however, the secondary form, associated with bacterial elastolytic activity and leukocyte‐derived elastases during inflammation, has been more commonly reported in the literature as linked to DS. (d) Physical examination of a patient with DS revealed numerous soft, oblong, and fleshy papules measuring 2−5 mm around the periorbital region, consistent with periorbital syringomas. These benign adnexal neoplasms originate from the eccrine sweat glands, and in patients with DS, they exhibit a higher rate of calcification, which may progress to calcinosis cutis and should be observed for potential changes. DS, Down syndrome.

**FIGURE 6:** Vascular and pigmentation disorders in individuals with DS. (a) Livedo reticularis on the anterior surface of the leg displays a typical net‐like pattern of reddish‐blue skin discoloration, often transient or permanent, usually following a benign course. (b) Infantile hemangioma on the right side of the patient's back, an angiogenesis‐dependent vascular tumor with a generally reduced risk of vascular anomalies in individuals with DS. (c) Acanthosis nigricans localized under the left armpit, presenting as dark velvety patches in the skin folds, a condition often associated with obesity and insulin resistance. (d) Widespread vitiligo manifesting as irregular white patches resulting from the loss of skin pigment, highlighting its association with autoimmune conditions commonly linked to DS. DS, Down syndrome.

## 4 Discussion

Among the 100 patients included in our study, 97 showed dermatological abnormalities. Xerosis was observed in 49% of patients, which is lower than the 85% reported by Carter et al. [13] but higher than the 33% found by Schepis et al. [14] and the 22% reported by Gunes Bilgili et al. [15]. Thin and sparse hair was noted in 48% of our patients, a finding not commonly reported in earlier studies, highlighting a unique aspect of our cohort. Dental caries were detected in 34% of our patients, consistent with the findings of Corder et al. [16], who also reported a prevalence of 34%. The observed differences in the prevalence of DS‐associated skin disorders across various studies are likely due to variations in patient age, recruitment methods, study design, geographical and environmental factors, and differences in healthcare access and diagnostic criteria. A detailed comparison of our findings with those of previous studies is presented in Table 6.

**TABLE 6:** Comparative analysis of dermatologic findings in patients with DS across different studies.

Year and first author	Country	Number of patients	Mean age (years)	M/F ratio	The most common dermatological findings (prevalence)
Carter, 1976 [13]	United States	214	Not include	128/86	Xerosis (85%), tinea pedis (76.6%), onychomycosis (67.8%)
Polenghi et al., 1990 [17]	Italy	96	Not include	Not include	Folliculitis (27%), alopecia areata (21%), psoriasis (8%)
Ercis et al., 1996 [18]	Türkiye	71	2.8	41/30	Palmar and plantar hyperkeratosis (40.8%), seborrheic dermatitis (30.9%), fissured tongue (20%)
Schepis et al., 2002 [14]	Italy	203	11.7	125/78	Xerosis (33%), folliculitis (21%), syringomas (12%)
Ferrando et al., 2003 [19]	Spain	416	Not include	Not include	Scrotal tongue (72.1%), atopic dermatitis including xerosis (63.4%), seborrhoeic dermatitis (21.6%)
Daneshpazhooh et al., 2007 [20]	Iran	100	11.2	47/53	Fissured tongue (28%), hypertrophy of tongue papillae (22%), premature graying (14%)
Araníbar et al., 2009 [21]	Chile	252	Not include	Not include	Keratosis pilaris (52%), xerosis (39%), seborrheic dermatitis (29%)
Gunes Bilgili, 2011 [15]	Türkiye	50	8.4	28/22	Xerosis (22%), Mongolian spot (22%), seborrheic dermatitis (16%)
Sureshbabu et al., 2011 [8]	India	95	12.0	59/36	Lichenification (52.6%), xerosis (43.2%), dental anomaly (35.8%)
Corder et al., 2017 [16]	United Arab Emirates	221	4	139/82	Dental caries (34%), eczema (14.2%), alopecia areata/totalis (2.7%)
Firsowicz et al., 2019 [22]	United States	243	13.1	115/128	Xerosis (25.5%), alopecia areata/totalis/universalis (21.0%), folliculitis (21%)
Gaber & Alghobashy, 2020 [23]	Egypt	50	Not include	28/22	Seborrheic dermatitis (65%), xerosis (42%), fissured tongue (30%)
Rork et al., 2020 [24]	United States	101	19.7	62/39	Folliculitis (30.7%), seborrheic dermatitis (26.7%), hidradenitis suppurativa (22.8%)
Our Study, 2024	Türkiye	100	6.37	46/54	Xerosis (49%), thin and sparse hair (48%), dental caries (34%)

Comparison of our study with previous research on dermatological findings in patients with DS. It highlights trends and variations in common skin conditions reported across different regions and periods. This comparative analysis underscores the consistent identification of dermatologic issues in patients with DS while reflecting regional and temporal differences, emphasizing the importance of regular and comprehensive dermatologic assessments for improved healthcare management in this population.

However, most dermatoses in DS patients are benign. Typical DS‐associated dermatoses include elastosis perforans serpiginosa, syringomas, milia‐like calcinosis cutis, multiple eruptive dermatofibromas, and transient myeloproliferative disorder [25]. In addition to syringomas, these conditions were not observed in the present study. We report a case of acrokeratosis verruciformis of Hopf, a genodermatosis characterized by verrucous papules on the dorsum of the hands and feet, which has not been previously documented in patients with DS.

Patients with DS are prone to early skin aging, including lentigines and wrinkles, as well as secondary eczematization associated with xerosis, which is attributed to altered skin barrier function, immune system variations, and associated conditions such as hypothyroidism. Approximately 70% of DS patients exhibit mild to moderate generalized xerosis, particularly affecting the ankles, knees, and legs. Related dermatological issues such as keratosis pilaris and hyperkeratosis of the extensor and palmoplantar surfaces are also common [26]. While keratosis pilaris was identified in 13% of the DS group, palmoplantar keratoderma and atopic dermatitis were observed in 6%, indicating a complex relationship between xerosis and these conditions. Despite initial expectations, the prevalence of atopic dermatitis was lower than anticipated when the Hanifin and Rajka criteria were applied [27]. Our findings highlight that, while xerosis cutis may not be highly specific, it carries notable significance for DS patients due to its higher prevalence and its association with other systemic and dermatological conditions. Managing xerosis is essential, as it can lead to increased discomfort, secondary complications, and a compromised skin barrier, making it a critical aspect of dermatological care in DS patients.

In our study, we observed that bacterial infections, predominantly folliculitis, had a prevalence of 11% among individuals with DS. Firsowicz et al. reported that folliculitis, acneiform eruptions, and pilonidal cysts are common in patients with DS, with a folliculitis prevalence of 21% [22]. Similarly, Rork et al. reported a higher prevalence of folliculitis (30.7%), HS (22.8%), and acne vulgaris (10.9%) [24].

The relationship between HS and DS was first reported by Dvorak et al. in 1977 [28]. Subsequent research indicated a younger onset age of onset of HS in DS patients and a higher prevalence of DS in the HS population [29], although one study found no link to HS severity [30]. Various studies have reported differing HS prevalences in DS patients, with Poizeau et al. at 15% [31], Sechi et al. at 24.4% [32], and Giovanardi et al. at 3.5% [33]. In our cohort, the prevalence of HS was 1%, possibly lower due to variations in sample size, demographics, genetics, environmental factors, and diagnostic criteria. This underscores the importance of regular HS screening and management in DS patients, as recommended annually by the US and Canadian Hidradenitis Suppurativa Foundations [34].

The genetic predisposition for HS and other follicular occlusion disorders in DS patients is linked to chromosome 21 trisomy, which results in elevated amyloid precursor protein (APP) levels. APP competes with the Notch receptor for gamma‐secretase processing, which is essential for HS pathogenesis, potentially disrupting Notch signaling and increasing the risk of follicular occlusion and HS. Additionally, DS patients’ heightened vulnerability to folliculitis may stem from inherent immunological weaknesses, marked by deficits in both cellular and humoral immunity [35, 36, 37].

In patients with DS, scabies is more often observed in its crusted form, likely due to cognitive delays impairing itch perception and immune system abnormalities such as T and B cell lymphopenia and impaired T cell proliferation [38]. In our cohort, the prevalence of scabies was significantly lower in individuals with DS than in the control group (*p* = 0.002), and males with DS were more affected than females (*p* = 0.047). Hypothetically, the lower prevalence of scabies in the DS group may be due to enhanced hygiene and healthcare supervision provided in rehabilitative care settings. These findings suggest that while individuals with DS may have a theoretical predisposition to more severe forms of scabies due to immunological and cognitive factors, the overall reduced prevalence in our cohort highlights the importance of controlled environments and proactive healthcare in mitigating the risk of infestation.

The additional copy of chromosome 21 in DS leads to the overexpression of certain genes, such as endostatin, which produces anti‐angiogenic factors that inhibit blood vessel formation and tumor growth [39]. Greene et al. found that individuals with DS have a reduced risk of vascular anomalies owing to the overexpression of several anti‐angiogenic proteins, including endostatin, DSCR1, and collagen XVIII [40]. In our cohort, hemangiomas were observed in 6% of individuals with DS compared with 3% in the control group (*p* > 0.05). This finding contrasts with the studies by Skinner et al., which suggested a reduced risk of vascular anomalies in DS due to elevated levels of anti‐angiogenic proteins [41]. Consistent with our study, a study conducted in the United States of 633 patients with DS found that these individuals have a lower risk of developing vascular anomalies than the general population [40].

In studies involving individuals with DS, the prevalence of cutis marmorata/livedo reticularis, which is often associated with congenital heart diseases, such as atrial and ventricular septal defects, was 8.8% in a cohort of 203 individuals, 12.6% in a cohort of 71 participants, and 8.4% in a cohort of 213 individuals, which are often associated with congenital heart diseases, such as atrial and ventricular septal defects [42]. In our study, vascular conditions such as cutis marmorata, livedo reticularis, and acrocyanosis were significantly more prevalent in the DS group (17%) compared to the control group (*p* < 0.001), with a higher prevalence observed in females compared to males (*p* < 0.001). Vascular instability could be a frequent cutaneous manifestation in individuals with DS, possibly due to poor peripheral circulation and an increased incidence of congenital heart disease.

CALM is commonly associated with genetic conditions, such as neurofibromatosis type 1, Legius syndrome, and McCune‐Albright syndrome [43]. In our cohort, however, these macules were observed more frequently in the DS group (15%) compared to the control group (4%) (*p* = 0.0008), and more frequently in males (18.5%) than in females (10.9%) (*p* = 0.009), suggesting a unique dermatological profile associated with DS. The higher prevalence of CALM in individuals with DS is thought to result from genetic and immunological variations inherent to DS, and the increased frequency in males compared to females may be influenced by hormonal factors.

In our study, the prevalence of vitiligo and alopecia areata (AA) was 3% in individuals with DS, although the difference was not statistically significant (both *p* > 0.05). Autoimmune diseases are more prevalent in this group, possibly due to the AIRE gene on chromosome 21 and enhanced interferon (IFN) receptor expression, which may predispose them to conditions such as vitiligo and AA [44]. This predisposition may lead to “super‐induction” of JAK/STAT signaling and IFN‐stimulated genes in individuals with DS. Additionally, IFN‐*γ* is considered central to the pathogenesis of both AA and vitiligo [45].

In our cohort of patients with DS, 7% had CTA. CTA is a circumscribed, noncicatricial form of alopecia typically found in the frontotemporal region, often detected in childhood or at birth, and is associated with various congenital conditions, including DS [46]. The literature on hair loss in individuals with DS primarily focuses on trace element deficiencies and autoimmunity, whereas reports on CTA remain underreported.

Prasher et al. found that 22 out of 50 children with DS exhibited nail changes, indicating a higher incidence of podiatric issues like pes planus and split toenails, emphasizing the need for specialized podiatric care [47]. In our cohort, 25% exhibited nail dystrophy, potentially due to factors such as hypothyroidism, infection susceptibility, and nutritional deficiencies.

The high prevalence of orofacial issues in individuals with DS, including low salivary pH, limited microbial diversity, frequent Candida species, and dental anomalies, significantly contributes to dental health challenges [48]. Our study revealed that these issues were notably more common than in the controls, featuring delayed tooth eruption (28%), fissured tongue (23%), dental caries (34%), and dental anomalies (22%) (all *p* < 0.0001). Corder et al. noted that dental caries occurs in 34.4% of individuals with DS, often due to prolonged bottle feeding and sugary diets [16]. Conversely, Deps et al. suggested that while many studies reported lower caries prevalence due to protective orofacial traits and salivary factors, some indicated higher rates, possibly due to inadequate dental care and poor dietary choices [49].

Using the Demirjian method, Van der Linden et al. demonstrated that dental development in children with DS is delayed compared to that in healthy children [50]. Al‐Maweri et al. reported a significantly higher prevalence of fissured tongue in children with DS (78%) compared to the control group, with an increased frequency observed in males and older age groups [51]. Similarly, our study found that fissured tongue was slightly more common in males than in females.

Dental anomalies are more prevalent in individuals with DS than in the general population, primarily because of the slow cellular growth rhythm and reduction in cell numbers affecting tooth development [52]. In our study, cheilitis was observed in 18% of individuals with DS, aligning with the findings of Scully et al., who reported a prevalence of 25% in the DS population. The increased prevalence of angular stomatitis in patients with DS is often associated with Candida albicans and is likely due to immune defects, mouth breathing, and orofacial abnormalities commonly observed in DS [53].

In our study, anetoderma was observed in 8% of individuals with DS. Kaplan et al. previously described anetoderma in patients with DS, hypothesizing a congenital malformation of elastic fibers [54]. The presence of the superoxide dismutase gene on chromosome 21, overexpression of COL6A1, and irregular type VI collagen arrangement in trisomy 21 may influence elastic fiber defects [55]. This may also be influenced by defective elastin synthesis, excessive elastolytic enzymes, and imbalances in matrix metalloproteinases (MMPs) and tissue inhibitors of metalloproteinases (TIMPs), which contribute to elastic fiber breakdown. Reduced expression of fibulin‐4, key to elastic fiber assembly, further underscores its importance in anetoderma pathogenesis [56, 57].

Upslanted palpebral fissures, epicanthal folds, and brachycephaly are nearly universal in individuals with DS, with other characteristic features present in 47%−82% of cases [58, 59]. In our study, the prevalence of epicanthal folds and upslanted palpebral fissures was 97% and brachycephaly was 91%, which is consistent with previous findings [60, 61]. Gender‐specific differences were noted, with brachycephaly and sandal gap being more common in males, highlighting the need for further research on these variations. Although the dismorphic features of DS are well‐documented, our findings on gender‐specific differences provide novel insights into the phenotypic variability of the condition and emphasize the need for further investigation. Additionally, the potential correlation between these dismorphic traits and dermatological findings, such as atopic dermatitis or keratosis pilaris, suggests a shared genetic basis that warrants further exploration to fully understand the comprehensive phenotypic expression in individuals with DS.

Karyotype analysis showed that trisomy 21 was present in 92% of the cases, mosaicism in 6%, and translocation in 2%. Similarly, high frequencies of mosaicism have been reported by Thomas et al. from Bangalore, with 86.6% trisomy, 7.7% translocation, and 5.8% mosaicism [62], and Jyothy et al., who also reported a high prevalence of mosaicism (7.69%) [63]. The variation in the frequency of cytogenetic anomalies may be due to differences in the time period, maternal age, and populations studied.

## 5 Conclusion

In conclusion, our comprehensive analysis of dermatological and dysmorphic features in individuals with DS identified prevalent characteristics such as xerosis, thin and sparse hair, and dental caries. Shortened leukocyte telomere length and impaired DNA repair mechanisms phenomena, associated with chromosomal anomalies on chromosome 21, and the resultant increase in oxidative stress are recognized contributors to the elevated prevalence of dermatological conditions in DS. Moreover, significant advancements in medical interventions, such as improvements in cardiac surgery, enhanced prevention of childhood infections, increased access to comprehensive healthcare, and improved psychosocial support, are also presumed to have contributed to this increase. Consistencies and variations in cytogenetic analyses compared to existing studies emphasize the need for ongoing research to fully delineate the spectrum of DS manifestations and enhance therapeutic strategies. An enhanced understanding of DS‐related skin disorders and comorbidities through continued research is crucial for improving patient outcomes, particularly for those who struggle to communicate their symptoms. All of this could lead to the establishment of specialized clinics for DS patients, improve the management of dermatological conditions, and encourage active participation in group‐living programs, thereby enhancing their overall well‐being.

## 6 Limitations

Despite conducting a power analysis prior to the study to determine an appropriate sample size, the cross‐sectional design and potential sample size limitations may restrict insights into the progression of conditions over time and fully represent the broader population. While we used standard diagnostic methods, the scope of some assessments may have led to underreporting certain conditions. Additionally, despite efforts to match the control group, some confounding factors, such as environmental factors and access to healthcare, could not be fully controlled.

## Conflicts of Interest

The authors declare no conflicts of interest.

## Data Availability

The data that support the findings of this study are available from the corresponding author upon reasonable request.

## References

[1] J. H. L. Down , “Observations on an Ethnic Classification of Idiots,” London Hospital Medical Reports 3, 1866: 259–262.

[2] J. Lejeune , M. Gautier , and R. Turpin , “Étude des Chromosomes Somatiques de Neuf Enfants Mongoliens [Study of Somatic Chromosomes From 9 Mongoloid Children],” Comptes Rendus Hebdomadaires des Séances de L'académie des Sciences 248, no. 11 (1959): 1721–1722.13639368

[3] N. J. Roizen and D. Patterson , “Down's Syndrome,” Lancet 361, no. 9365 (2003): 1281–1289, 10.1016/S0140-6736(03)12987-X.12699967

[4] I. Açikbaş , A. Tomatir , B. Akdağ , and A. Koksal , “Retrospective Analysis of Live Birth Prevalence of Children With Down Syndrome in Denizli,” Turkey Genetics and Molecular Research 11, no. 4 (2012): 4640–4645, 10.4238/2012.September.10.1.23079965

[5] D. Türkbay , F. E. Canpolat , T. Derme , N. Altuğ , and Y. Yılmaz , “The Birth Prevalence of Selected Major Congenital Anomalies: Six‐Year's Experience in a Tertiary Care Maternity Hospital,” Turkish Pediatric Archives 55, no. 4 (2020): 393–400, 10.14744/TurkPediatriArs.2020.36097.PMC775035133414657

[6] S. E. Antonarakis , R. Lyle , E. T. Dermitzakis , A. Reymond , and S. Deutsch , “Chromosome 21 and Down Syndrome: From Genomics to Pathophysiology,” Nature Reviews Genetics 5, no. 10 (2004): 725–738, 10.1038/nrg1448.15510164

[7] S. E. Antonarakis , B. G. Skotko , M. S. Rafii , et al., “Down Syndrome,” Nature Reviews Disease Primers 6, no. 1 (2020): 9, 10.1038/s41572-019-0143-7.PMC842879632029743

[8] R. Sureshbabu , R. Kumari , S. Ranugha , R. Sathyamoorthy , C. Udayashankar , and P. Oudeacoumar , “Phenotypic and Dermatological Manifestations in Down Syndrome,” Dermatology Online Journal 17, no. 2 (2011): 3.21382286

[9] M. Contaldo , R. Santoro , A. Romano , et al., “Oral Manifestations in Children and Young Adults With Down syndrome: A Systematic Review of the Literature,” Applied Sciences 11, no. 12 (2021): 5408, 10.3390/app11125408.

[10] T. J. Pikora , J. Bourke , K. Bathgate , K. R. Foley , N. Lennox , and H. Leonard , “Health Conditions and Their Impact Among Adolescents and Young Adults With Down Syndrome,” PLoS ONE 9, no. 5 (2014): e96868, 10.1371/journal.pone.0096868.24818963 PMC4018436

[11] V. Desingu , A. Adapa , S. Kumar , and S. Devi , “Dental Anomalies in Down Syndrome Individuals: A Review,” Journal of Science in Dentistry 9, no. 1 (2019): 6–8, 10.5005/jp-journals-10083-0902.

[12] J. McGowan‐Jordan , R. Hastings , and S. Moore , “Re: International System for Human Cytogenetic or Cytogenomic Nomenclature (ISCN): Some Thoughts, by T. Liehr,” Cytogenetic and Genome Research 161, no. 5 (2021): 225–226, 10.1159/000516655.34407535

[13] D. M. Carter , “Alopecia Areata and Down Syndrome,” Archives of Dermatology 112, no. 9 (1976): 1397–1400, 10.1001/archderm.1976.01630340015003.134671

[14] C. Schepis , C. Barone , M. Siragusa , and C. Romano , “An Updated Survey on Skin Conditions in Down Syndrome,” Dermatology 205, no. 3 (2002): 234–238, 10.1159/000065859.12399669

[15] S. G. Bilgili , N. Akdeniz , A. S. Karadag , S. Akbayram , O. Calka , and H. U. Ozkol , “Mucocutaneous Disorders in Children With Down Syndrome: Case‐controlled Study,” Genetic Counseling (Geneva, Switzerland) 22, no. 4 (2011): 385–392.22303799

[16] J. P. Corder , F. J. S. Al Ahbabi , H. S. Al Dhaheri , and F. Chedid , “Demographics and Co‐Occurring Conditions in a Clinic‐Based Cohort With Down Syndrome in the United Arab Emirates,” American Journal of Medical Genetics Part A 173, no. 9 (2017): 2395–2407, 10.1002/ajmg.a.38338.28686324

[17] M. M. Polenghi , F. Piattoni , G. B. Orsini , et al., “Dermatologic Disorders in Down syndrome (Abstract),” American Journal of Medical Genetics 7(Suppl.) (1990): 324.

[18] M. Ercis , I. Inanir , N. Elmaci , N. Gunes , and O. Ozturk , “Dermatological Manifestations of 71 Down Syndrome Children Admitted to a Clinical Genetics Unit,” Clinical Genetics 50, no. 4 (1996): 317–320, 10.1111/j.1399-0004.1996.tb02381.x.9007317

[19] J. Ferrando and C. Escobar , “Incidencia de Patología Dermatológica en los Pacientes del Centre Mèdic Down de la Fundació Catalana Síndrome de Down,” Revista Médica Internacional del Síndrome de Down 7 (2003): 39–43.

[20] M. Daneshpazhooh , M. Radmanesh , and S. A. Hashemi , “Mucocutaneous Findings in 100 Children With Down Syndrome,” Pediatric Dermatology 24, no. 3 (2007): 317–320, 10.1111/j.1525-1470.2007.00412.x.17542890

[21] L. Araníbar , B. Villagrán , D. Merino , E. Hernández , and M. Espinoza , “Dermatologic Disorders in Patients With Down Syndrome in Santiago, Chile,” Journal of the American Academy of Dermatology 60, no. 3 (2009): AB145, 10.1016/j.jaad.2008.11.639.

[22] M. Firsowicz , I. J. Frieden , L. F. Eichenfield , and B. A. Drolet , “Follicular Occlusion Disorders in Down Syndrome Patients,” Pediatric Dermatology 36, no. 5 (2019): 616–620, 10.1111/pde.14012.31626333

[23] M. A. Gaber and M. S. A. Alghobashy , “Mucocutaneous Findings in Down Syndrome,” Menoufia Medical Journal 33, no. 3 (2020): 1007–1010, 10.4103/mmj.mmj_405_18.

[24] J. F. Rork , L. McCormack , K. Lal , K. Wiss , and L. Belazarian , “Dermatologic Conditions in Down Syndrome: A Single‐Center Retrospective Chart Review,” Pediatric Dermatology 37, no. 5 (2020): 811–816, 10.1111/pde.14214.32519435

[25] R. Fölster‐Holst , T. Rohrer , and A.‐M. Jung , “Dermatological Aspects of the S2k Guidelines on Down Syndrome in Childhood and Adolescence,” JDDG: Journal Der Deutschen Dermatologischen Gesellschaft 16, no. 12 (2018): 1289–1295, 10.1111/ddg.13665.30300491

[26] J. Casals , N. S. Baldrich , E. Rozas‐Muñoz , and R. Monserrat , “The Pathophysiology and Management of Xerosis and Mouth Conditions in Patients With Trisomy 21,” Revista Médica Internacional Sobre El Síndrome De Down 21, no. 3 (2017): 46–50, 10.1016/J.SDENG.2017.10.001.

[27] C. Schepis , C. Barone , M. Siragusa , and C. Romano , “Prevalence of Atopic Dermatitis in Patients With Down Syndrome: A Clinical Survey,” Journal of the American Academy of Dermatology 36, no. 6 (1997): 1019–1021, 10.1016/s0190-9622(97)80294-0. Pt 1.9204075

[28] V. C. Dvorak , R. K. Root , and R. R. MacGregor , “Host‐Defense Mechanisms in Hidradenitis Suppurativa,” Archives of Dermatology 113, no. 4 (1977): 450–453.848973

[29] G. Denny and M. J. Anadkat , “Hidradenitis Suppurativa (HS) and Down Syndrome (DS): Increased Prevalence and a Younger Age of Hidradenitis Symptom Onset,” Journal of the American Academy of Dermatology 75, no. 3 (2016): 600–601, 10.1016/j.jaad.2016.04.045.27543219

[30] J.‐C. Hernández‐Rodríguez , G.‐F. Osorio‐Gómez , J. Ortiz‐Álvarez , J.‐A. Lebrón‐Martín , J. Conejo‐Mir , and J.‐J. Pereyra‐Rodríguez , “Hidradenitis Suppurativa and Down Syndrome in a Single‐Centre Sample: A Cross‐Sectional Study,” Australasian Journal of Dermatology 63, no. 3 (2022): e231–e237, 10.1111/ajd.13872.35567765

[31] F. Poizeau , E. Sbidian , C. Mircher , et al., “Prevalence and Description of Hidradenitis Suppurativa in Down Syndrome: A Cross‐Sectional Study of 783 Subjects,” Acta Dermato‐Venereologica 99, no. 3 (2019): 351–352, 10.2340/00015555-3095.30460373

[32] A. Sechi , A. Guglielmo , A. Patrizi , et al., “Disseminate Recurrent Folliculitis and Hidradenitis Suppurativa Are Associated Conditions: Results From a Retrospective Study of 131 Patients With Down Syndrome and a Cohort of 12,351 Pediatric Controls,” Dermatology Practical & Conceptual 9, no. 3 (2019): 187–194, 10.5826/dpc.0903a03.31384491 PMC6659610

[33] G. Giovanardi , A. Chiricozzi , L. Bianchi , et al., “Hidradenitis Suppurativa Associated With Down Syndrome Is Characterized by Early Age at Diagnosis,” Dermatology 234, no. 1‐2 (2018): 66–70, 10.1159/000487799.29689550

[34] A. Garg , N. Malviya , A. Strunk , et al., “Comorbidity Screening in Hidradenitis Suppurativa: Evidence‐Based Recommendations From the US and Canadian Hidradenitis Suppurativa Foundations,” Journal of the American Academy of Dermatology 86, no. 5 (2022): 1092–1101, 10.1016/j.jaad.2021.01.059.33493574 PMC8298595

[35] O. Berezovska , C. Jack , A. Deng , N. Gastineau , G. W. Rebeck , and B. T. Hyman , “Notch1 and Amyloid Precursor Protein Are Competitive Substrates for Presenilin1‐Dependent Gamma‐Secretase Cleavage,” Journal of Biological Chemistry 276, no. 32 (2001): 30018–30023, 10.1074/jbc.M008268200.11408475

[36] J. Blok , M. Jonkman , and B. Horváth , “The Possible Association of Hidradenitis Suppurativa and Down Syndrome: Is Increased Amyloid Precursor Protein Expression Resulting in Impaired Notch Signaling the Missing Link?,” British Journal of Dermatology 170, no. 6 (2014): 1375–1377, 10.1111/bjd.12887.24506173

[37] B. C. Melnik and G. Plewig , “Impaired Notch‐MKP‐1 Signaling in Hidradenitis Suppurativa: An Approach to Pathogenesis by Evidence From Translational Biology,” Experimental Dermatology 22, no. 3 (2013): 172–177, 10.1111/exd.12098.23489419

[38] R. Murugaiyan , K. L. Sengottian , and K. Karthikeyan , “Crusted Scabies Presenting as Palmoplantar Psoriasis in Down's Syndrome,” Indian Dermatology Online Journal 6, no. 2 (2015): 140–141, 10.4103/2229-5178.153025.25821745 PMC4375766

[39] T. S. Zorick , Z. Mustacchi , S. Y. Bando , et al., “High Serum Endostatin Levels in Down syndrome: Implications for Improved Treatment and Prevention of Solid Tumours,” European Journal of Human Genetics: EJHG 9, no. 11 (2001): 811–814, 10.1038/sj.ejhg.5200721.11781696

[40] A. K. Greene , S. Kim , G. F. Rogers , S. J. Fishman , B. R. Olsen , and J. B. Mulliken , “Risk of Vascular Anomalies With Down Syndrome,” Pediatrics 121, no. 1 (2008): e135–e140, 10.1542/peds.2007-1316.18166531

[41] R. Skinner , “Angiogenesis: How Down's Syndrome Protects,” Nature Reviews Cancer 9, no. 9 (2009): 649–650, 10.1038/nrc2687.

[42] V. Madan , J. Williams , and J. T. Lear , “Dermatological Manifestations of Down's Syndrome,” Clinical and Experimental Dermatology 31, no. 6 (2006): 741–749, 10.1111/j.1365-2230.2006.02164.x.16901300

[43] K. N. Shah , “The Diagnostic and Clinical Significance of Café‐Au‐Lait Macules,” Pediatric Clinics of North America 57, no. 5 (2010): 1131–1153, 10.1016/j.pcl.2010.07.002.20888463

[44] M. Giménez‐Barcons , A. Casteràs , P. Armengol Mdel , et al., “Autoimmune Predisposition in Down Syndrome May Result From a Partial Central Tolerance Failure Due to Insufficient Intrathymic Expression of AIRE and Peripheral Antigens,” Journal of Immunology (Baltimore, MD: 1950) 193, no. 8 (2014): 3872–3879, 10.4049/jimmunol.1400223.25217160

[45] C. Ryan , K. Vellody , L. Belazarian , and J. F. Rork , “Dermatologic Conditions in Down Syndrome,” Pediatric Dermatology 38, no. 1 (2021): 49–57, 10.1111/pde.14731.34418156

[46] M. Yamazaki , R. Irisawa , and R. Tsuboi , “Temporal Triangular Alopecia and a Review of 52 Past Cases,” Journal of Dermatology 37, no. 4 (2010): 360–362, 10.1111/j.1346-8138.2010.00817.x.20507407

[47] V. P. Prasher , L. Robinson , V. H. Krishnan , and M. C. Chung , “Podiatric Disorders Among Children With Down Syndrome and Learning Disability,” Developmental Medicine and Child Neurology 37, no. 2 (1995): 131–134, 10.1111/j.1469-8749.1995.tb11982.x.7851669

[48] S. C. Möhlhenrich , P. Schmidt , S. Chhatwani , et al., “Orofacial Findings and Orthodontic Treatment Conditions in Patients With Down Syndrome—A Retrospective Investigation,” Head & Face Medicine 19, no. 1 (2023): 15, 10.1186/s13005-023-00362-5.37149612 PMC10163777

[49] T. D. Deps , G. L. Angelo , C. C. Martins , S. M. Paiva , I. A. Pordeus , and A. C. Borges‐Oliveira , “Association Between Dental Caries and Down Syndrome: A Systematic Review and Meta‐Analysis,” PLoS ONE 10, no. 6 (2015): e0127484, 10.1371/journal.pone.0127484.26086498 PMC4472226

[50] M. S. van der Linden , S. Vucic , D. J. F. van Marrewijk , and E. M. Ongkosuwito , “Dental Development in Down Syndrome and Healthy Children: A Comparative Study Using the Demirjian Method,” Orthodontics & Craniofacial Research 20, no. 2 (2017): 65–70, 10.1111/ocr.12139.28207178

[51] S. A. Al‐Maweri , B. Tarakji , G. A. Al‐Sufyani , H. M. Al‐Shamiri , and G. Gazal , “Lip and Oral Lesions in Children With Down Syndrome. A Controlled Study,” Journal of Clinical and Experimental Dentistry 7, no. 2 (2015): e284–e288, 10.4317/jced.52283.26155347 PMC4483338

[52] O. A. Cuoghi , F. Topolski , L. Perciliano de Faria , et al., “Prevalence of Dental Anomalies in Permanent Dentition of Brazilian Individuals With Down Syndrome,” Open Dentistry Journal 10 (2016): 469–473, 10.2174/1874210601610010469.27733874 PMC5045970

[53] C. Scully , W. van Bruggen , P. Diz Dios , B. Casal , S. Porter , and M. F. Davison , “Down Syndrome: Lip Lesions (Angular Stomatitis and Fissures) and Candida Albicans,” British Journal of Dermatology 147, no. 1 (2002): 37–40, 10.1046/j.1365-2133.2002.04741.x.12100182

[54] H. Kaplan , E. Lacentre , and S. Carabelli , “Alteraciones del Tejido Elástico en Pacientes con Síndrome de Down [Changes in the Elastic Tissue of Patients With Down's Syndrome],” Medicina Cutanea Ibero‐Latino‐Americana 10, no. 2 (1982): 79–84.6218349

[55] C. S. von Kaisenberg , B. Brand‐Saberi , B. Christ , S. Vallian , F. Farzaneh , and K. H. Nicolaides , “Collagen Type VI Gene Expression in the Skin of Trisomy 21 Fetuses,” Obstetrics and Gynecology 91, no. 3 (1998): 319–323, 10.1016/s0029-7844(97)00697-2.9491853

[56] S. Weinstein and W. Piette , “Cutaneous Manifestations of Antiphospholipid Antibody Syndrome,” Hematology/Oncology Clinics of North America 22, no. 1 (2008): 67–vi, 10.1016/j.hoc.2007.10.011.18207066

[57] T. Gambichler , L. Reininghaus , M. Skrygan , et al., “Fibulin Protein Expression in Mid‐Dermal Elastolysis and Anetoderma: A Study of 23 Cases,” Acta Dermato‐Venereologica 96, no. 5 (2016): 708–710, 10.2340/00015555-2340.26775654

[58] K. L. Jones , “Down Syndrome,” in Smith's Recognizable Patterns of Human Malformation (6th ed., Elsevier Saunders, 2006), p. 7.

[59] C. J. Epstein , C. R. Scriver , A. L. Beaudet , W. S. Sly , and D, Valle , eds, The Metabolic & Molecular Bases of Inherited Disease (McGraw‐Hill, 2001). 1223–1256.

[60] L. Devlin and P. J. Morrison , “Accuracy of the Clinical Diagnosis of Down Syndrome,” Ulster Medical Journal 73, no. 1 (2004): 4–12.15244118 PMC2475449

[61] M. P. Kava , M. S. Tullu , M. N. Muranjan , and K. M. Girisha , “Down Syndrome: Clinical Profile From India,” Archives of Medical Research 35, no. 1 (2004): 31–35, 10.1016/j.arcmed.2003.06.005.15036797

[62] I. M. Thomas , S. Rajangam , and S. Hegde , “Cytogenetic Investigations in Down Syndrome Patients & Their Parents,” Indian Journal of Medical Research 96 (1992): 366–371.1289249

[63] A. Jyothy , K. S. Kumar , G. N. Rao , et al., “Cytogenetic Studies of 1001 Down Syndrome Cases From Andhra Pradesh, India,” Indian Journal of Medical Research 111 (2000): 133–137.10935320

